The article "Pantoea agglomerans: An Elusive Contributor to Chronic Obstructive Pulmonary Disease Exacerbation" was published in 2021. Journal: Cureus.

# Pantoea agglomerans: An Elusive Contributor to Chronic Obstructive Pulmonary Disease Exacerbation

**DOI:** 10.7759/cureus.18562

**Published:** 2021-10-07

**Authors:** Binav Shrestha, Nabin K C, Chhabilal Bastola, Tahmina Jahir, Ruby Risal, Shivani Thapa, Danilo Enriquez, Frances Schmidt

**Affiliations:** 1 Pulmonary Medicine, Interfaith Medical Center, Brooklyn, USA; 2 Internal Medicine, Interfaith Medical Center, Brooklyn, USA

**Keywords:** chronic obstructive pulmonary disease, copd, pantoea agglomerans, bacteremia, copd exacerbation, gram-negative bacteria

## Abstract

The ubiquitously present gram-negative bacteria *Pantoea agglom*erans is not a commonly known human pathogen. Recently, increasing recognition of the species as a human pathogen has led to controversy as limited documented cases of *P.* *agglomerans* bacteremia and infections have been reported in the literature, with most cases reported among immunocompromised patients or the pediatric population. Here, we present the case of a 54-year-old female with *P. agglomerans* and *Enterococcus faecium *bacteremia along with chronic obstructive pulmonary disease.

## Introduction

The genus Pantoea, gram-negative rods with yellow pigmentation belonging to the Erwiniaceae family, has been reported to cause opportunistic infections in immunocompromised patients. Only a few cases of spontaneous *Pantoea agglomerans* bacteremia have been reported, mostly among pediatric, hospitalized, immunocompromised, or cancer patients [1-3]. Although it is present in the soil, plant surfaces, human excreta, vegetables, and fruits, it is known to jump kingdoms and cause a clinical spectrum of diseases ranging from diarrhea, sepsis, arthritis, osteomyelitis, synovitis, urinary tract infections, pneumonia, to septic shock in humans [3-5]. The impact of *P. agglomerans* bacteremia remains largely unknown in chronic respiratory disorders such as chronic obstructive pulmonary disease (COPD).

## Case presentation

A 54-year-old female with a history of (Global Initiative for Chronic Obstructive Lung Disease stage 3 and group D) multiple COPD exacerbations and one with endotracheal intubation, without home oxygen, 16 pack-year cigarette smoking, and marijuana abuse came to the emergency department for worsening shortness of breath with nonproductive cough, myalgia, and watery diarrhea for three days. Other systems were normal.

At presentation, she was afebrile, with a heart rate of 112 beats per minute, respiratory rate of 30 breaths per minute, and saturation of 95-98% on 3 L of oxygen on nasal cannula. Bilateral wheezing with few crepitations was noted on the bilateral bases of the lungs. The rest of the examination was unremarkable. Labs at the time of admission showed leukocytosis of 15.6 × 10^9^/L (reference range: 4.5-11 × 10^9^/L) with a left shift of neutrophils at 88.3% and relative lymphopenia at 4.5% (0.7 × 10^9^/L). The chemistry panel was near-normal with the following findings: Na+/K+ of 139/3.9 mmol/L, Cl- of 97 mmol/L, elevated HCO_3_ of 32 mEeq/L, and normal anion gap of 10. Blood urea nitrogen (BUN)/creatinine ratio was 13.0/0.66 mg/dL, with a slightly elevated glucose level of 173 mg/dL. Furthermore, calcium, phosphorus, and magnesium levels were 8.9 mg/dL, 5.3 mg/dL, and 1.9 mg/dL, respectively. Liver function tests showed total bilirubin of 0.5 mg/dL, aspartate transaminase of 14 U/L, alanine transaminase of 13 U/L, alkaline phosphatase of 119 U/L, total protein of 5.9 g/dL, albumin of 3.7 m/dL, and elevated bicarbonate of 35.7 mEq/L. Moreover, urine toxicology was positive for cannabinoids. Polymerase chain reaction (PCR) test for coronavirus disease 2019 (COVID-19) was negative, and influenza, mycoplasma, and *Legionella* antigen tests were also negative. Lactate dehydrogenase was elevated at 322 U/L (reference range: 125-220 U/L), and total creatine kinase was 43 U/L. D-dimer was 414 ng/mL with a normal coagulation profile with prothrombin time (PT) of 12.8 seconds and activated partial thromboplastin time of 31.3 seconds. PT/international normalized ratio was 1.09. Chest X-ray showed hyperinflation with mild perihilar congestion without any evidence of consolidation and no significant changes compared with the prior study. Computed tomography (CT) without contrast revealed mildly hyperinflated lungs with mild emphysematous changes predominating in the apices, along with scattered small areas of fibrotic changes. No convincing lung consolidation or acute infiltrate pleural effusion was noted, with normal mediastinum, heart size, and unremarkable hila with pericardial effusion (Figure 1).

The article "Pantoea agglomerans: An Elusive Contributor to Chronic Obstructive Pulmonary Disease Exacerbation" was published in 2021. Journal: Cureus.

**Figure 1:** CT chest showing no consolidation and emphysematous changes due to COPD. Incidental finding of small GGO in the left lower lobe. CT: computed tomography; COPD: chronic obstructive pulmonary disease; GGO: ground-glass opacities

Arterial blood gas (ABG) on 2 L of oxygen via nasal cannula showed pH of 7.299, pCO_2_ of 75 mmHg, pO_2_ of 72.9 mmHg, HCO_3-_ of 35 mmol/L, and oxygen saturation of 96%. Sequential Organ Failure Assessment (SOFA) score was less than 2 (less than 9 implies <33.3% mortality), and PaO_2_/FiO_2_ ratio was 260. She was admitted to the hospital for acute hypoxic and hypercapnic respiratory failure secondary to COPD exacerbation and was started on methylprednisolone along with albuterol and ipratropium nebulization and intravenous ceftriaxone and azithromycin. Her clinical course worsened on days two and three of admission with tachypnea, fatigue, as well as occasional and multiple episodes of desaturation of up to 86% on 2 L of oxygen via a nasal cannula. She was switched to bilevel positive airway pressure (BiPAP) with inspiratory positive airway pressure/expiratory positive airway pressure of 15/5 mmHg, with a respiratory rate of 15 breaths per minute and FiO_2_ of 40% due to worsening respiratory status. Two repeat PCR tests for COVID-19 were negative. Blood culture sent at the time of admission grew two organisms later identified as *E. faecium* and *P. agglomerans*.

She was fairly compliant with BiPAP, and on day four of admission, she started improving clinically and reported feeling comfortable on 2-3 L of oxygen via a nasal cannula with on and off BiPAP (approximately six to seven hours) during the night. Her ABG on BiPAP with FiO_2_ of 40% oxygen also showed improvement with pH of 7.339, pCO_2_ of 63.7 mmHg, pO_2_ of 87.2 mmHg, HCO_3-_ of 33 mmol/L, and oxygen saturation of 97%. Antibiotic sensitivity analysis of E. faecium and P. agglomerans revealed that both were sensitive to ceftriaxone. Therefore, ceftriaxone and azithromycin were continued for five days, with a continued tapering dose of steroids.

Of note, another set of blood cultures sent on the day of admission and on days two and three during deterioration showed no growth in the subsequent follow-up. On day six of admission, the patient improved significantly and was discharged home with home oxygen therapy with proper instructions regarding the medication and oxygen therapy. On the two-week follow-up at the medical clinic, she reported remarkable improvement in respiratory symptoms and was using oxygen during nights with the occasional need for inhaler use.

## Discussion

*Pantoea* species are yellow-pigmented, Gram-negative, rod-shaped, aerobic bacteria belonging to the Erwiniaceae family. Based on shared protein homologs, it was previously classified in the Enterobacteriaceae family along with *Klebsiella*, *Escherichia*, *Salmonella*, and *Enterobacter *[6-8]. It is commonly isolated from plant surfaces, seeds, fruits, and animal/human feces. Humans get exposed by ingestion of infected plants or thorn pricks. However, It can also cause opportunistic infections in humans, especially when the immune system is impaired. This case report aims to investigate the clinical features, pathogenesis, and treatment course of *P. agglomerans* bacteremia in a patient with COPD and bring attention to the association of this rare bacterium with COPD. *P. agglomerans* is a rare cause of blood, wound, and respiratory and urinary infections which usually present as fever, chills, and disseminated diseases such as septic arthritis, endophthalmitis, endocarditis, and osteomyelitis in the setting of bacteremia. Spontaneous infection can occur in an immunocompromised host. Typically, the bacteria have low virulence and a mild clinical course, with timely antibiotic initiation resulting in a favorable outcome.

The article "Pantoea agglomerans: An Elusive Contributor to Chronic Obstructive Pulmonary Disease Exacerbation" was published in 2021. Journal: Cureus.

Ubiquitous in the environment, *P. agglomerans* is found naturally in cotton and has been speculated as a possible pathological contribution in byssinosis and hypersensitivity pneumonitis (HP) [9,10]. In Eastern Poland, it has been identified as the most important cause of HP [11]. It is also postulated that inhaled *P. agglomerans* endotoxins elicit pathologic processes similar to cotton dust, resulting in the activation of alveolar macrophages and secretion of mediators such as interleukin-1, tumor necrosis factor (TNF), and prostaglandins. These mediators lead to the accumulation of platelets in pulmonary capillaries triggering acute and chronic inflammation associated with byssinosis. These changes subsequently result in bronchoconstriction, reduced forced expiratory volume in the first second, reduced diffusing capacity of the lung for carbon monoxide, and increased airway reactivity, which leads to significant respiratory symptoms [10]. The dominant presence of *P. agglomerans* (as high as 31.25%) has been reported in respiratory samples of immunocompromised patients presenting with respiratory symptoms, raising the possibility of its effect among patients with poorly controlled COPD with chronic exposure to steroids similar to our patient [12].

Spontaneous bacteremia with *P. agglomerans* has been associated with gastroesophageal reflux disease, active malignancy, and end-stage renal disease patients [13]. In our case, the patient had multiple hospitalizations due to COPD exacerbations leading to multiple and prolonged doses of steroids. Hence, therapeutic use of steroids in COPD can act as a double-edged sword; on one hand, helping acute exacerbation, while, on the other hand, leading to opportunistic infections such as *P. agglomerans*. Most previously documented cases of *P. agglomerans* bacteremia have been reported in clinical settings associated with central venous line, osteomyelitis, urinary tract infection, or isolated from abscess cavities. It should be noted that only about 20% of reported case reports and case series were able to isolate *Pantoea* species in two sets of blood cultures. It is our understanding that while *Pantoea *bacteremia may be transient, its potential for clinical deterioration could not be ignored, as seen in our case of clinical deterioration after days two to three of admission. In concordance with previous literature findings of transient bacteremia and significant clinical improvement after antibiotics, our case proves that early diagnosis and proper antibiotic use can prevent potential complications [14]. Of note, most reported *Pantoea *species infections are sensitive to broad-spectrum antibiotics. Other clinically relevant species of *Pantoea* have been reported such as *P. brenneri* in the urethra, *P. dispersa* in central line infections, *P. gavinae* and *P. calida* among formula feeding infants, and *P. conspicua* occasionally isolated in blood [15-17]. All of the species have been documented to infect both immunocompetent and immunocompromised individuals. Except for the occasional grave clinical course, most clinical entities described in regards to *P. agglomerans* are amenable to the treatment by appropriate antibiotics and supportive management, as seen in our case [18]. In addition to its association with many diseases, it is being evaluated for its potential role as immunopotentiators (IP-PA1) causing increased expression of cytokines such as TNF and causing macrophage activation and reversal of immunosuppression after chemotherapy. They are also being investigated for therapeutic use against cancers such as melanoma and allergic conditions [19].

The article "Pantoea agglomerans: An Elusive Contributor to Chronic Obstructive Pulmonary Disease Exacerbation" was published in 2021. Journal: Cureus.

According to a 2014 systematic review, 15.1-30% of the U.S. population suffers from GERD. Some of these patients can present with atypical symptoms such as cough, asthma, laryngitis, or chest pain. Although our patient did not report a history of underlying GERD, it is worth noting that COPD and GERD are commonly associated with *P. agglomerans*, possibly acting synergistically and worsening outcomes in COPD [20]. Of note, GERD is very prevalent and may contribute to lung pathologies such as COPD and interstitial lung disease [20-22]. Widespread occurrence and potential of inhalational transmission make *P. agglomerans* a possible cause of COPD exacerbations [23]. To our knowledge, this is the first case report speculating the possibility of *P. agglomerans* as a potential contributing factor for the pathology of COPD. In complex diseases with multifactorial pathophysiology such as COPD where a small trigger can have fatal consequences, the potential causes which could be easily treated should be further investigated. Bacteremia with *P. agglomerans* and *E. faecium *co-infection in colon cancer has been reported previously in the literature, but our case report describes spontaneous bacteremia with *P. agglomerans* and *E. faecium* in an individual presenting with COPD exacerbation without previously documented risk factors [24].

The article "Pantoea agglomerans: An Elusive Contributor to Chronic Obstructive Pulmonary Disease Exacerbation" was published in 2021. Journal: Cureus.

## Conclusions

The epidemiology and clinical significance of *P. agglomerans* are still largely unknown in COPD. *P. agglomerans* can cause bacteremia in COPD patients which can be treated successfully with proper antibiotics. Further large-scale studies are needed to evaluate its potential role in exacerbation and its prognostic value in COPD.
